The article "Immunoglobulin G4+ B‐cell receptor clones distinguish immunoglobulin G 4‐related disease from primary sclerosing cholangitis and biliary/pancreatic malignancies" was retracted in 2022. Reasons: errors in the results or conclusions; concerns about the images.

# Immunoglobulin G4^+^ B‐cell receptor clones distinguish immunoglobulin G 4‐related disease from primary sclerosing cholangitis and biliary/pancreatic malignancies

**DOI:** 10.1002/hep.28568

**Published:** 2016-06-08

**Authors:** Marieke E. Doorenspleet, Lowiek M. Hubers, Emma L. Culver, Lucas J. Maillette de Buy Wenniger, Paul L. Klarenbeek, Roger W. Chapman, Frank Baas, Stan F. van de Graaf, Joanne Verheij, Thomas M. van Gulik, Eleanor Barnes, Ulrich Beuers, Niek de Vries

**Affiliations:** ^1^ Amsterdam Rheumatology and Immunology Center, Department of Clinical Immunology & Rheumatology, Academic Medical CenterAmsterdamThe Netherlands; ^2^ Department of Genome AnalysisAcademic Medical CenterAmsterdamThe Netherlands; ^3^ Department of Gastroenterology & Hepatology and Tytgat Institute for Liver and Intestinal ResearchAcademic Medical CenterAmsterdamThe Netherlands; ^4^ Translational Gastroenterology UnitJohn Radcliffe HospitalOxfordUnited Kingdom; ^5^ NDM Oxford University, Oxford Martin School, Oxford UniversityOxfordUnited Kingdom; ^6^ Department of PathologyAcademic Medical CenterAmsterdamThe Netherlands; ^7^ Department of SurgeryAcademic Medical CenterAmsterdamThe Netherlands; ^8^ Present address: Department of OphthalmologyVU Medical CenterAmsterdamThe Netherlands

## Abstract

Immunoglobulin G4 (IgG4)‐related disease (IgG4‐RD) of the biliary tree and pancreas is difficult to distinguish from sclerosing cholangitis and biliary/pancreatic malignancies (CA). An accurate noninvasive test for diagnosis and monitoring of disease activity is lacking. We demonstrate that dominant IgG4^+^ B‐cell receptor (BCR) clones determined by next‐generation sequencing accurately distinguish patients with IgG4‐associated cholangitis/autoimmune pancreatitis (n = 34) from those with primary sclerosing cholangitis (n = 17) and CA (n = 17). A novel, more affordable, and widely applicable quantitative polymerase chain reaction (qPCR) protocol analyzing the IgG4/IgG RNA ratio in blood also achieves excellent diagnostic accuracy (n = 125). Moreover, this qPCR test performed better than serum IgG4 levels in sensitivity (94% vs. 86%) and specificity (99% vs. 73%) and correlates with treatment response (n = 20). *Conclusions*: IgG4^+^ BCR clones and IgG4/IgG RNA ratio markedly improve delineation, early diagnosis, and monitoring of IgG4‐RD of the biliary tree and pancreas. (Hepatology 2016;64:501‐507)

**Abbreviations**
AIP: autoimmune pancreatitis
ANOVA: analysis of variance
AUC: area under the curve
BCR: B‐cell receptor
CCA: cholangiocarcinoma
CA: biliary/pancreatic malignancies
cDNA: complementary DNA
CP: chronic pancreatitis
HISORt: histology, imaging, serology, other organ involvement, response to treatment
IAC: IgG4‐associated cholangitis
IgG4: immunoglobulin G4
IgG4‐RD: IgG4‐related disease
IQR: interquartile range
NGS: next‐generation sequencing
PSC: primary sclerosing cholangitis
qPCR: quantitative polymerase chain reaction
ROC: receiver operating characteristic
SSC: secondary sclerosing cholangitis
sIgG4: serum IgG4
ULN: upper limit of normal

Immunoglobulin G4 (IgG4)‐related disease (IgG4‐RD) is a multiorgan inflammatory disease that frequently affects the biliary tree (IgG4‐associated cholangitis; IAC) and pancreas (autoimmune pancreatitis; AIP).^1^, ^2^ Its pathogenesis is enigmatic. Clinical presentations of IAC and AIP show striking similarities to those of primary/secondary sclerosing cholangitis (PSC/SSC), cholangiocarcinoma (CCA), chronic pancreatitis (CP) of other cause, and pancreatic carcinoma (PC). No single diagnostic test can accurately diagnose biliary and pancreatic manifestations of IgG4‐RD. Elevated serum IgG4 (sIgG4) levels are neither sensitive nor specific for IgG4‐RD^3^, ^4^, ^5^, ^6^; up to 30% of IAC/AIP patients have normal sIgG4 levels. Furthermore, increased sIgG4 levels are present in 10%‐20% of patients with PSC and biliary/pancreatic malignancies (CA). Given that these conditions are far more prevalent than IgG4‐RD, the positive predictive value of sIgG4 levels is poor when only moderately elevated. Composite scores, such as the HISORt (histology, imaging, serology, other organ involvement, response to treatment) criteria,^7^, ^8^ are regarded as diagnostic standards, and a consensus on diagnostic pathological features is available.^9^ Still, misdiagnosis is common, and 1 in 3 patients with IgG4‐RD has undergone major interventions because of suspected malignancy before diagnosis.^7^, ^8^ Therefore, ready‐to‐use tests with high diagnostic accuracy are urgently needed. Moreover, because relapse after tapering of immunosuppressive therapy occurs in 50% of IAC/AIP patients,^10^ biomarkers for treatment response and disease activity are highly desired.

The article "Immunoglobulin G4+ B‐cell receptor clones distinguish immunoglobulin G 4‐related disease from primary sclerosing cholangitis and biliary/pancreatic malignancies" was retracted in 2022. Reasons: errors in the results or conclusions; concerns about the images.

Recently, we identified dominant IgG4^+^ B‐cell receptor (BCR) clones in peripheral blood of 6 patients with active IAC, but not in healthy or disease controls, using next‐generation sequencing (NGS).^11^ This novel technique enables identification of IgG4^+^ clones within the BCR repertoire. Of note, the same clones were encountered in the inflamed tissue.^11^ Consequently, this test could represent a novel diagnostic tool. Here, we aimed to validate our previous findings in a prospective, case‐control study. Furthermore, we evaluated the diagnostic accuracy of a novel, more affordable, and widely applicable test based on quantitative polymerase chain reaction (qPCR) and compared it with that of sIgG4 levels. Moreover, we evaluated whether the qPCR test may be used to monitor treatment response.

## Patients and Methods

### STUDY SUBJECTS

Consecutive patients meeting the HISORt diagnostic criteria for IAC^7^ and/or AIP^8^ were prospectively enrolled in this case‐control study. In line with HISORt criteria, three diagnostic pathways were possible: (1) patient had undergone a pancreatic/biliary resection for a presumed malignancy or a core biopsy showing diagnostic pathological features of AIP/IAC (group A)^7^, ^8^; (2) patient showed classical imaging for AIP in combination with elevated sIgG4 levels of >1.4 g/L (group B)^7^, ^8^; and (3) patient had suspicion of pancreatic disease and/or strictures of bile ducts together with two or more of the following: elevated sIgG4 levels, suggestive pancreatic imaging findings, other organ involvement, and/or bile duct biopsy with >10 IgG4^+^ B cells/high‐power field in combination with marked improvement of pancreatic morphology/biliary strictures and biochemical parameters upon 4 weeks of corticosteroid treatment (group C).^7^, ^8^ Moreover, patients had active disease as confirmed by laboratory and/or radiographical findings. Patients were naïve to immunosuppressive treatment or experienced a recurrence of symptoms with laboratory/radiographic changes requiring a higher dose of immunosuppression. Controls consisted of patients with PSC and CA. PSC patients were diagnosed according to the 2009 European Association for the Study of the Liver Clinical Practice Guidelines “Management of cholestatic liver diseases,” based on serological findings (cholestatic serum liver test profile; supportive: atypical perinuclear antineutrophil cytoplasmic antibody), combined with typical findings of multifocal strictures and dilatations on magnetic resonance cholangiopancreaticography and/or endoscopic retrograde cholangiopancreaticography and exclusion of causes for SSC.^12^ Diagnosis in patients with CA was confirmed by histopathology (biopsy or resection material) and/or cytology (brush cytology or fine needle aspiration biopsy) together with imaging. In addition, consecutive patients with chronic pancreatitis diagnosed according to the guidelines of the American Pancreatic Association based on suggestive history, abnormal pancreas physiology, and abnormal imaging findings^13^ were included. Control patients did not use immunosuppressive treatment. Enrollment took place at the Department of Gastroenterology and Hepatology at the Academic Medical Center (University of Amsterdam) in Amsterdam, The Netherlands, and at the John Radcliffe Hospital (Oxford University) in Oxford, United Kingdom. The study was approved by the local medical ethical committees (MEC AMC 10/007, NL 31142.018.09; Oxford research ethics RECA 10/H0604/51); all study subjects gave written informed consent before inclusion, and the study was performed according to the principles of the Declaration of Helsinki.

The article "Immunoglobulin G4+ B‐cell receptor clones distinguish immunoglobulin G 4‐related disease from primary sclerosing cholangitis and biliary/pancreatic malignancies" was retracted in 2022. Reasons: errors in the results or conclusions; concerns about the images.

### SERUM IgG4 LEVELS

sIgG4 levels (upper limit of normal [ULN] = 1.4 g/L) were measured in 122 patients by automated nephelometry in the local laboratory (using BN ProsPec Siemens in Amsterdam and BNII Siemens in Oxford). For 3 patients, a sIgG4 level was only measured after start of treatment, not at time of RNA collection.

### PERIPHERAL BLOOD SAMPLING AND HANDLING

Peripheral blood was collected in PAXGene Blood RNA tubes (catalog no. 762165; PreAnalytiX, Breda, The Netherlands) at the Academic Medical Center in Amsterdam and in Tempus Blood RNA tubes (catalog no. 4342792; Life Technologies, Paisley, UK) at the John Radcliffe Hospital in Oxford and handled according to manufacturer's instructions. Simultaneously or at least within 1 week, serum was collected for IgG4 measurement. Processing of blood RNA tubes was performed by a trained technician masked for the origin of the samples or outcome of the sIgG4 levels. In a similar fashion, the person performing the data analysis (M.D.) was blinded. Complementary DNA (cDNA) was synthesized from 1,000 ng of total RNA input using Superscript III RT (Invitrogen Life Technologies, Carlsbad, CA).

### LINEAR AMPLIFICATION AND NGS

The linear amplification protocol has been extensively described earlier.^14^ Samples were prepared for sequencing according to the manual for amplicon sequencing and sequenced on a Roche Genome Sequencer FLX (Titanium platform; Roche Diagnostics, Almere, The Netherlands). For each sample 10,000 BCR_heavy_ sequences were analyzed. NGS visualizes expanded BCR clones as a deviation in the repertoire because the BCR sequence they carry is determined more frequently than low abundant BCR sequences and thus account for a relatively large proportion of all the sequences found. Moreover, it is not unlikely that plasmacytoid cells are identified in peripheral blood; these cells produce increased amounts of BCR messenger RNA, producing a comparable deviation in the repertoire as expanded B cells. For clarity, we will use the term “dominant clone” to denote these clones.

### qPCR

IgG and IgG4 primers for qPCR were designed to specifically amplify sequences that encode the constant region of the heavy chain of the receptor and according to common standards for primer design (Supporting Fig. S1). Additionally, the following rules were applied: (1) two different reverse primers were designed, one for all possible IgG subtypes and one specific for the IgG4 subtype, and (2) the two reverse primers were designed on virtually the same position to allow comparable conditions. After optimization, this resulted in one universal *forward* primer (5′‐GCTGCCTGGTCAAGGACTAC‐3′), one generic IgG *reverse* primer (5′‐TCTTGTCCACCTTGGTGTTG‐3′), and one specific IgG4 *reverse* primer (5′‐CTACGTTGCAGGTGTAGGTCTTC‐3′). Duplicate qPCR reactions were performed in a 10‐μL total volume in the presence of 10 pmol of the forward and reverse primers, cDNA from 50 ng RNA input, and 5 μL of SensiFAST SYBR Lo‐ROX reagent (catalog no. BIO‐94005, Bioline; GC Biotech, Alphen aan den Rijn, Netherlands) for 40 cycles (95°C for 2 minutes, 40 cycles [95°C for 5 seconds, 60°C for 10 seconds, and 72°C for 20 seconds], followed by a melting curve [95°C for 5 seconds, 65°C for 1 minute, and 97°C continuous]), using the LightCycler 480 system (Roche Diagnostics, Almere, The Netherlands). Both for IgG and IgG4, the starting concentrations in the sample were calculated using LinRegPCR software^15^ and used to calculate the percentage of IgG^+^ RNA molecules that were IgG4^+^. Thus, the more expanded IgG4^+^ clones were present in blood, the higher the percentage IgG4 RNA message of total IgG RNA message.

The article "Immunoglobulin G4+ B‐cell receptor clones distinguish immunoglobulin G 4‐related disease from primary sclerosing cholangitis and biliary/pancreatic malignancies" was retracted in 2022. Reasons: errors in the results or conclusions; concerns about the images.

### BIOINFORMATICS PIPELINE AND DATA ANALYSIS

The bioinformatics pipeline used to obtain the BCR sequences was described in detail^16^ and contains four modules: MID sorting; identification of gene segments; CDR3 detection; and removal of artefacts. Immunoglobulin isotype homology was determined using the National Center for Biotechnology Information's open‐access Web tool BLASTn (megablast algorithm) and reference sequences for the human immunoglobulin heavy‐chain constant regions, allowing a sequence homology >97%.^16^

### STATISTICAL ANALYSIS

Following criteria for (non)parametric analysis, values are expressed as mean ± SD or median and interquartile range (IQR). Differences between groups were analyzed using Student *t* test, Mann‐Whitney *U* test, one‐way analysis of variance (ANOVA), Kruskal‐Wallis test of ranks, or χ^2^ test, where appropriate. A receiver operating characteristic (ROC) curve was used to determine cut‐off values for diagnosis of IgG4‐RD. Diagnostic accuracy was expressed in terms of sensitivity and specificity rates with 95% confidence intervals. Graphpad Prism (GraphPad Prism (version 6; GraphPad Software Inc., La Jolla, CA) and PASW Statistics software (version 22; SPSS, Inc., Chicago, IL) were used to perform statistical analyses. Two‐sided *P* values of <0.05 were considered statistically significant. This study was performed in agreement with the Standards for Reporting of Diagnostic Accuracy.

The article "Immunoglobulin G4+ B‐cell receptor clones distinguish immunoglobulin G 4‐related disease from primary sclerosing cholangitis and biliary/pancreatic malignancies" was retracted in 2022. Reasons: errors in the results or conclusions; concerns about the images.

## Results

A total of 50 IgG4‐RD patients meeting the HISORt criteria for IAC and/or AIP were prospectively included at two departments of Gastroenterology and Hepatology in Amsterdam and Oxford between December 2011 and December 2015. In total, 15 patients were included in HISORt group A, 13 in HISORt group B, and 22 in HISORt group C. Forty‐eight patients with PSC, 27 with CA, and 10 patients with CP served as disease controls. Patient characteristics are described in Supporting Tables S1 and S2.

Sequencing the BCR repertoire (n = 34 IgG4‐RD patients; n = 34 controls) revealed multiple dominant IgG4^+^ BCR clones within the IgG^+^ repertoire of IgG4‐RD patients (Fig. 1A) compared to disease controls (Fig. 1B). This is reflected in a strikingly higher percentage of IgG^+^ BCR clones being IgG4^+^ (Fig. 1C), a greater fraction of the IgG^+^ repertoire being taken in by IgG4^+^ BCRs (Fig. 1D), and a higher rank of the most dominant IgG4^+^ BCR clone in IgG4‐RD patients compared to controls (Fig. 1E), confirming our previous findings.^11^

**Figure 1:** **BCR repertoire in IgG4‐related disease and disease controls** (A,B) scatterplot showing the IgG^+^ repertoires in 34 patients suffering from IgG4‐RD (IRD01‐IRD34; A) and disease controls (B), consisting of PSC (PSC01‐PSC17; n = 17) and CA (CA01‐CA17; n = 17). Every dot represents a unique IgG^+^ clone. IgG4^+^ clones are marked in red. (C) Bar chart showing the distribution of IgG1+, IgG2+, IgG3+, and IgG4‐positive clones of all IgG+ clones within the repertoire in IgG4‐RD, PSC, and CA. (D) Bar chart showing the part of the repertoire taken up by IgG4^+^ BCRs versus IgG4^‐^ BCRs in IgG4*‐*RD, PSC, and CA. (E) Ranks of the most dominant IgG4^+^ clones within the IgG^+^ repertoire in IgG4‐RD, PSC, and CA (*P* < 0.0001).

In order to distinguish IgG4‐RD patients from disease controls on a widely available platform, a qPCR protocol was developed that estimates the fraction of total IgG RNA that encodes IgG4 (qPCR test). Using this qPCR test in blood samples of a Dutch discovery cohort—consisting of 15 IgG4‐RD patients, 7 PSC patients, and 8 CA patients (including patients published earlier for NGS analysis only^11^)—resulted in clear differences between the three groups (Supporting Fig. S2). The cutoff for the qPCR test was determined at 5% of all IgG^+^ RNA molecules being IgG4^+^ using an ROC curve. Subsequently, the cut‐off value was validated in additional cohorts from two clinical sites (Dutch cohort: 26 IAC/AIP, 11 PSC, and 19 CA patients; British cohort: 9 IAC/AIP and 30 PSC; Supporting Fig. S2). The overall sensitivity and specificity of all cohorts combined was 94.0% and 98.7%, respectively (χ^2^, 109; *P* = 1*10^−29^; Fig. 2A). The area under the curve (AUC) value of 0.991 (Fig. 2B) indicated excellent accuracy. Post‐hoc analysis showed a cut‐off value ranging from 3.5% to 6% had the best clinical utility indices, depending on the aim to avoid false positives or negatives. Additional subanalysis in 40 IgG4‐RD patients with pancreatic involvement and 10 CP patients was performed, and showed comparable results for both BCR repertoire analysis as well as the qPCR test (Supporting Fig. S3).

The article "Immunoglobulin G4+ B‐cell receptor clones distinguish immunoglobulin G 4‐related disease from primary sclerosing cholangitis and biliary/pancreatic malignancies" was retracted in 2022. Reasons: errors in the results or conclusions; concerns about the images.

**Figure 2:** **qPCR test in IgG4‐RD and disease controls** (A) dot plot showing the percentage specific IgG4 RNA molecules of total IgG RNA molecules in 50 IgG4‐RD patients, 48 PSC patients, and 27 patients suffering from CA. The red dotted line delineates the cut‐off value of 5%; ^***^ *P* < 0.001. (B) ROC curve of the qPCR test for the prediction of IgG4‐RD (50 cases vs. 75 controls). The arrow points to the cut‐off value and denotes this value. (C) Before‐after dot plot showing the qPCR test values in 20 IgG4‐RD patients at baseline, and 4 and 8 weeks after high‐dose corticosteroid therapy. The red dotted line delineates the cut‐off value of 5%; ^***^ *P* < 0.001.

Comparing the findings of the qPCR test to a well‐used marker, sIgG4, the latter showed a sensitivity and specificity for sIgG4 of 85.7% and 73.3% (χ^2^, 41; *P* = 9*10^−11^; Supporting Fig. S2), respectively. Because sIgG4 is part of the diagnostic criteria for IgG4‐RD (HISORt groups B and C), we performed a subanalysis on the different diagnostic subgroups. This showed that the sensitivity of sIgG4 in patients in whom sIgG4 was not part of the diagnostic criteria was lower (group A: sensitivity, 67%; χ^2^, 9; *P* = 0.005; group B: sensitivity, 100%; χ^2^, 25; *P* = 5*10^−7^; group C: sensitivity, 91%; χ^2^, 28; *P* = 1*10^−7^), whereas the qPCR test performed equally in all three groups (group A: sensitivity, 87%; χ^2^, 69; *p* = 9*10^−13^; group B: sensitivity, 100%; χ^2^, 81; *P* = 1*10^−14^; group C: sensitivity, 96%; χ^2^, 86; *P* = 5*10^−19^; Supporting Fig. S4).

Subanalysis of follow‐up samples in 20 Dutch IAC/AIP patients 4 and 8 weeks after start of corticosteroid therapy revealed an IgG4 RNA decrease from 20.3% ± 13.4% of total IgG RNA (mean ± SD) before treatment to 5.8% ± 2.2% after 4 weeks and 1.9% ± 0.8% after 8 weeks (Fig. 2C; *P* < 0.0001). All patients responded well and showed clinical improvement with resolution of symptoms, together with a decrease of biochemical markers (Supporting Fig. S5).

In conclusion, analysis in 34 IgG4‐RD cases and 34 disease controls using NGS confirms our former findings^11^ that both the number and size of dominant clones are increased in peripheral blood of IgG4‐RD patients, compared to disease controls. The rank of the most dominant IgG4^+^ BCR clone clearly discriminates between IgG4‐RD and disease controls. A simple qPCR test in 50 patients and 85 controls showed comparable diagnostic properties and, in addition, can be used to monitor treatment response.

The article "Immunoglobulin G4+ B‐cell receptor clones distinguish immunoglobulin G 4‐related disease from primary sclerosing cholangitis and biliary/pancreatic malignancies" was retracted in 2022. Reasons: errors in the results or conclusions; concerns about the images.

## Discussion

The current study in 135 patients confirms recent findings^11^ that the presence of dominant IgG4^+^ BCR clones in peripheral blood determined by NGS clearly distinguishes patients with IgG4‐RD of the biliary tree and pancreas from disease controls with similar clinical presentation, such as pancreatobiliary cancer or PSC. Our novel qPCR test adds to these findings by providing an accurate and affordable test for the diagnosis of IgG4‐RD and monitoring of treatment response.

The observation that a quarter of the IgG^+^ BCR repertoire is taken up by IgG4^+^ sequences in IgG4‐RD led us to speculate that IgG4^+^ RNA, rather than the released protein, may be used to diagnose IgG4‐RD early and accurately. Therefore, we developed a simple‐to‐use qPCR test that appeared to correlate better with diagnosis than sIgG4 titers, currently the best test available in peripheral blood. Given that the majority of patients in our cohort were included in the absence of a resection or core biopsy, a relatively high proportion of IgG4‐RD patients had elevated sIgG4 levels. A subanalysis in the diagnostic groups revealed that sensitivity of sIgG4 levels in the resection/core biopsy group in whom sIgG4 did not play a diagnostic role was limited (67%), in line with other cohorts. This cannot only be explained by the fact that a definite diagnosis of IgG4‐RD in patients with normal sIgG4 needs histology, but it is also known that sIgG4 levels are lower in IgG4‐RD patients after resection for a presumed malignancy given that at least part of the cells producing the sIgG4 are removed. In disease control groups with PSC and CA, however, sIgG4 levels, but not IgG4 RNA, were elevated, contributing to low specificity of sIgG4 levels. This highlights again the usefulness of this qPCR test as a simple and accurate test for diagnosis and monitoring in an otherwise difficult‐to‐diagnose disorder.

Three IgG4‐RD patients with elevated sIgG4 had a qPCR score below the threshold of 5%, and repertoire analysis performed in 2 patients showed no dominant IgG4^+^ clones among the top 10 of IgG^+^ clones. One of the 3 patients was diagnosed with CCA 32 months after fulfilling the HISORt criteria for IgG4‐RD. This emphasizes the need for even more accurate diagnostic criteria than the HISORt criteria and the potential of the presented qPCR test.

The article "Immunoglobulin G4+ B‐cell receptor clones distinguish immunoglobulin G 4‐related disease from primary sclerosing cholangitis and biliary/pancreatic malignancies" was retracted in 2022. Reasons: errors in the results or conclusions; concerns about the images.

Although most PSC patients with elevated sIgG4 values had normal IgG4/IgG RNA ratio, their qPCR scores were, on average, higher than in PSC patients with normal sIgG4. It has been suggested that PSC patients with elevated sIgG4 levels have worse clinical outcome in terms of disease severity and time to transplantation compared to PSC patients with normal levels.^18^ Whether this also holds true for the IgG4/IgG RNA ratio needs further investigation, but the only false‐positive qPCR score in the PSC group belonged to a patient with severe fibrosis and chronic inflammation on liver histology. Moreover, 1 PSC patient was identified with elevated sIgG4 and an infiltrate of >30 IgG4^+^ B cells on liver biopsy, a phenomenon that is regularly observed in liver explants of PSC patients with a severe disease course.^19^ Indeed, the qPCR score of 3.93% in this patient was relatively high. The patient was recently transplanted because of decompensated cirrhosis and progressive liver failure.

Both our previous and current findings on IgG4^+^ BCR clones are supported by a recent study confirming that plasmablasts are present in blood of IgG4‐RD patients.^20^ Our previous observation that a vast majority of IgG4‐RD patients were “blue‐collar workers” chronically exposed to solvents, industrial gases, or oil products^21^ (confirmed by actual data of Supporting Table S2) supports our view of specific immune responses underlying IgG4‐RD and may explain the advanced age and male predominance of IgG4‐RD patients.^21^ Moreover, the abnormal response to food and animal antigens in IgG4‐RD deserves attention.^22^

In conclusion, identification of dominant IgG4^+^ BCR clones in IgG4‐RD has enabled us to develop an affordable qPCR test, which may allow accurate diagnosis of IgG4‐related disease of the biliary tree and pancreas.

Author names in bold designate shared co‐first authorship.

## Supporting information

Additional Supporting Information may be found at onlinelibrary.wiley.com/doi/10.1002/hep.28568/suppinfo.

Supporting Information
